# HDAC Inhibition Decreases the Expression of EGFR in Colorectal Cancer Cells

**DOI:** 10.1371/journal.pone.0018087

**Published:** 2011-03-25

**Authors:** Chia-Wei Chou, Ming-Shiang Wu, Wei-Chien Huang, Ching-Chow Chen

**Affiliations:** 1 Department of Pharmacology, College of Medicine, National Taiwan University, Taipei, Taiwan; 2 Division of Gastroenterology, Department of Internal Medicine and Primary Care Medicine, College of Medicine, National Taiwan University and National Taiwan University Hospital, Taipei, Taiwan; 3 Graduate Institute of Cancer Biology, China Medical University, Taichung, Taiwan; 4 Center for Molecular Medicine, China Medical University Hospital, Taichung, Taiwan; University of Hong Kong, Hong Kong

## Abstract

Epidermal growth factor receptor (EGFR), a receptor tyrosine kinase which promotes cell proliferation and survival, is abnormally overexpressed in numerous tumors of epithelial origin, including colorectal cancer (CRC). EGFR monoclonal antibodies have been shown to increase the median survival and are approved for the treatment of colorectal cancer. Histone deacetylases (HDACs), frequently overexpressed in colorectal cancer and several malignancies, are another attractive targets for cancer therapy. Several inhibitors of HDACs (HDACi) are developed and exhibit powerful antitumor abilities. In this study, human colorectal cancer cells treated with HDACi exhibited reduced EGFR expression, thereby disturbed EGF-induced ERK and Akt phosphorylation. HDACi also decreased the expression of SGLT1, an active glucose transporter found to be stabilized by EGFR, and suppressed the glucose uptake of cancer cells. HDACi suppressed the transcription of EGFR and class I HDACs were proved to be involved in this event. Chromatin immunoprecipitation analysis showed that HDACi caused the dissociation of SP1, HDAC3 and CBP from EGFR promoter. Our data suggested that HDACi could serve as a single agent to block both EGFR and HDAC, and may bring more benefits to the development of CRC therapy.

## Introduction

EGFR (also known as ErbB-1/HER1), which belongs to the ErbB family of receptor tyrosine kinases, comprises an extracellular ligand-binding domain, a single hydrophobic transmembrane domain and a cytoplasmic tyrosine kinase-containing domain [1]. Ligand binding induces homo- or hetero-dimerization of receptor and subsequent activation of the pathways including Ras/Raf/MEK/ERK and PI3K/PDK1/Akt [1]. Most of colorectal cancer (CRC) is characterized with overexpression of epidermal growth factor receptor (EGFR) and predicted with high risk of metastasis and recurrence [2]. Targeting EGFR seems to be a promising approach for the CRC treatment. Indeed, cetuximab, a human-mouse chimeric IgG1 antibody binds to the external domain of the EGFR, has been approved by FDA in 2004 for the treatment of metastatic colorectal cancer [3]. After that, a fully humanized antibody, panitumumab, is also approved to treat CRC [4]. However, accumulating evidences demonstrate that the effects of targeting EGFR in colorectal cancer are largely limited due to the status of KRAS mutation [5]. The KRAS mutants bypass EGFR to activate the Ras/Raf/MEK/ERK signals, and significantly weaken the therapeutic effect of cetuximab [6]. Examination of KRAS status is now a prerequisite for the use of cetuximab [7]. Although ∼60% of CRC patients expressed wild-type KRAS but only half of them benefits from cetuximab. Therefore, the KRAS status is not the only determinant for the efficacy of EGFR target therapy [8]. Therefore, treatment with a broad spectrum of genetic backgrounds is urgently needed and would benefit most patients irresponsive to cetuximab-based therapies.

Although EGFR is a receptor tyrosine kinase and delivers signals after ligand conjugation, its prosurvival effect can be independent to kinase activity. For example, mice lacking EGFR are embryonic lethal but those harboring kinase-inactive mutants only exhibit some epithelial defects [9], [10]. In addition, loss of EGFR kinase activity decelerates cell proliferaiton but loss of its expression ruins the glucose uptake and leads to cell death [11]–[13]. Therefore, inhibition of EGFR expression may be a better strategy for CRC therapy.

Histone deacetylases (HDACs) which removes the acetyl groups from histone to silence the gene transcription are highly expressed in various tumors [14], [15]. HDACs have become one of the emerging targets for cancer therapy, and HDAC inhibitors (HDACi) show promising anticancer activities [15]. Among various HDACi, SAHA (Vorinostat) had been successfully approved for the treatment of cutaneous T cell lymphoma (CTCL). HDAC family can be subdivided into four classes and the class I HDACs, which includes HDAC1, HDAC2, HDAC3 and HDAC8, have been reported to be highly expressed in colon cancer [16]. The pro-proliferative effects of HDACs are connected to the transcriptional repression of cdk-inhibitor, p21, and knockdown of HDAC 1, 2 and 3 reduced the growth of several colon cancer cells [17]. Therefore, HDAC may serve as a potential target for CRC therapy, and SAHA had entered clinical trials for the treatment of CRC [18].

In this study, we demonstrated that the EGF signaling in KRAS mutant cell lines, HCT116 and SW480, was disrupted by HDACi through transcriptional repression of EGFR expression, indicating that HDACi served as a single agent to block EGFR and HDAC simultaneously. Loss of EGFR partially contributed to the cytotoxic effect of HDAC inhibitors. In addition, the expression of SGLT1, an active glucose transporter which is stabilized by EGFR, was also decreased by HDACi and led to the reduction of glucose uptake in colon cancer cells. The mechanism underlying the transcriptional repression of EGFR by HDACi was involved with the histones hypoacetylation and the dissociation of SP1, HDAC3 and CBP from EGFR promoter. Our data suggested that HDACi could serve as a single agent to concurrently block both EGFR and HDAC, and may bring benefits to the CRC patients with a broader range of genetic backgrounds.

## Materials and Methods

### Ethics Statement

All patient-derived specimens were collected and archived under protocols approved by Institutional Research Board of National Taiwan University Hospital and supported by the National Science Council, Taiwan. A full verbal explanation of the study was given to all participants. They consented to participate on a voluntary basis.

### Materials

TSA was purchased from Sigma and SAHA were obtained from Merck. The Myc-tagged HDAC1, 2 and 3 were provided by Dr. WM Yang (NCHU, Taiwan). Antibodies specific for EGFR, p21, HDAC3, and actin were purchased from Santa Cruz Biotechnology. Anti–Ac-histone H3, H4, and Sp1 antibodies were obtained from Upstate. Anti-SGLT1 antibody was purchased from Abcam.

### Cell culture

HCT-116 (from Van Dyke MW, M.D. Anderson) and SW480 (from TH Leu, NCKU) human colon carcinoma cells were cultured in DMEM supplemented with 10% fetal bovine serum; A431 (human epidermoid carcinoma cells) and MDA-MB-468 (human breast adenocarcinoma cells) obtained from ATCC were maintained in RPMI supplemented with 10% FCS.

### RNA isolation, RT-PCR and real time PCR

Total RNA was isolated from HCT116 cell using Trizol reagent (Life Technology). Reverse transcription reaction was performed using 2 µg of total RNA, reverse transcribed into cDNA using oligo dT primer. cDNA was subjected to RT-PCR and amplified 30 cycles using two oligonucleotide primers derived from published EGFR or GAPDH sequence, including 5′- TGGAGCTACGGGGTGACCGT-3′ and 5’-GGTTCAGAGGCTGATTGTGAT-3′ (EGFR), 5′-AAGCCCATCACCATCTTC-CAG-3′ and 5′-AGGGGCCATCCACA-GTCTTCT-3′(GAPDH) and 5′-TGAC-GGGGTCACCCACACTGTGCCCATCTA-3′ and 5′-CTAGAAGCATTTGCG-GGGACGATGGAGGG-3′(Actin). The PCR products were subjected to 1.2% agarose gel electrophoresis and visualized by ethidium bromide staining. Real time PCR was performed with cDNA samples using the ABI Prism 7900 Sequence Detection System (Applied Biosystems, Foster City, CA). Primers were as follows: EGFR (forward primer, 5′-TTCCTCCCAGTGCCTGAAT-3′ reverse primer, 5′-GGTTCAGAGGCTGAT-TGTGAT-3′); Actin (forward primer, 5′-CCAACCG-CGAGAAGATGA-3′; reverse primer, 5’-TCCATCACGATGCCAGTG-3’). The data were normalized by the Actin housekeeping gene detection.

### Cell proliferation

For growth inhibition analysis, HCT116 cells were seeded at a density of 3×10^3^ cells per well in 96-well plates. After seeding, the growth medium was replaced with medium containing indicated concentration of TSA. After 3 days, cell growth was measured using 3-(4,5-dimethylthiazol-2-yl)-2,5-diphenyltetrazolium bromide (Sigma, St. Louis, MO) colorimetric method. Cell cycle was determined by flow cytometry using a propidium iodide stain buffer and analyzed on a BD FACS Calibur cytometer with Cellquest software.

### Measurement of Intracellular Glucose

Prior to harvesting, adherent cultures of control and TSA-treated cells in DMEM containing 1 or 4.5 mg/ml glucose were washed twice with cold phosphate- buffered saline (PBS) and then lysed with ion-freeH_2_O for 5 min on ice. The glucose content was measured with D-glucose measurement kit (GAHK-20, Sigma-Aldrich, St. Louis, MO) according to the manufacturer’s protocol.

### Transient transfection and luciferase activity assay

The EGFR promoter plasmid containing a firefly luciferase was transiently transfected into HCT116 cells with Arrestin transfection reagent. Briefly, 0.9 µg of plasmid DNA, 0.1 µg of Renilla luciferase, and 5 uL transfection reagents were mixed, and the transfection protocol was carried out according to the manufacturer’s instructions (Promega). Six hours after transfection, the cells were cultured in the normal complete medium for another 16 h. Then, the transfected cells were subjected to luciferase assay. The firefly luciferase activity was normalized to that of the Renilla luciferase.

### Preparation and infection of shHDAC-expressing lentivirus

Briefly, 6 µg pCMV-dR8.91, 3 µg pMD2.G, and 9 µg pLKO-shLuciferase, pLKO-shHDAC1, pLKO-shHDAC2 or pLKO-shHDAC3 were cotransfected into HEK293T cells using Lipofectamine 2000 (Invitrogen). The supernatants containing infectious shLuciferase, shHDAC1, shHDAC2 or shHDAC3 lentivirus were collected on day 3 after transfection and stored at −80°C. For lentivirus infection, 2×10^5^ HCT116 cells were infected with shLuciferase, shHDAC1, shHDAC2 or shHDAC3 lentivirus at a multiplicity of infection (MOI) of 1.

### Patients and specimen preparation

Specimens of tumor tissue and adjacent normal tissue of colon were obtained from 14 patients who have been pathologically diagnosed colon cancer and underwent surgical resection at the National Taiwan University Hospital. Tissue specimens were ground, then sonicated in the lysis buffer (50 mM Tris-HCl, pH 7.4, 1 mM EGTA, 150 mM NaCl, 5% Triton X-100) with protease inhibitors. The samples were microcentrifuged to remove the larger debris and subjected to western analysis.

### Chromatin immunoprecipitation assay

Cells were treated with 5 µM SAHA for 6 h and cross-linked with 1.42% formaldehyde for 15 min. Cells in two 10-cm dishes were scraped in 1 ml of cold PBS, centrifuged, and lysed in 1 mL of IP buffer (150 mM NaCl, 50 mM Tris-HCl, pH 7.5, 5 mM EDTA, 0.5% Nonidet P-40, and 1% Triton X-100) containing protease inhibitors (1 mM phenylmethylsulfonyl fluoride, 1 µM leupeptin and 1 µM aprotinin). The nuclear pellet was resuspended in IP buffer and sonicated to shear chromatin. The sonicated lysates were immunoprecipited with antibodies against SP1, AcH3, AcH4, H3K4Me2, CBP and HDAC3, respectively and the immune complexes were recovered with protein A-Sepharose (Roche). The immunoprecipitated DNA and input DNA were extracted by incubating with 100 µl of 10% Chelex (Bio-Rad), boiling to reverse the cross-link, and centrifuging to remove Chelex slurry. Real-time PCR was performed with the purified DNA using the following primers: A: 5′- GTGAAAAACCCCACCGTTC-3′ and 5′- TCTGAAGGGGAGCAACCTTA-3′; B: 5′-AAGCTTCCGCGAGTTTCC-3′ and 5′- GAGGCTAAGTGTCCCACTGC-3′; C: 5′- ACCCTGGCACAGATTTGG-3′ and 5′- TGAGGAGTTAATTTCCGAGAGG-3’; D: 5′-CCAGTATTGATCGGGAGAGC-3′ and 5′- TTCCTCCAGAGCCCGACT-3′; E: 5′-CTGAGGAAGGAACCCAAAAA-3′ and 5′-GGGAGGTCCTCTCAGAA AGC-3′.

### Statistical analysis

Triplicate experiments were performed and results are presented as mean±SE. The two- tailed Student’s t test was used to calculate the statistical significance between group

## Results

### HDAC inhibitors disrupt the EGF signaling via silencing EGF receptor (EGFR) expression

To examine the antitumor effect of HDACi in colorectal cancer, KRAS wild type (WiDR and HT29) and KRAS mutant cells (HCT116 and SW480) were treated with SAHA or cetuximab for 48 hours, and cell viability was measured. SAHA reduced the survival of these cells in a dose-dependent manner (Fig. 1A), suggesting the independence of the KRAS status on the antitumor activity of HDACi. In contrast, cetuximab had little effect on the cell viability (Fig. 1A). This result is consistent with the previous study that colorectal cancer cells treated with cetuximab were killed more efficiently by antibody-dependent cellular cytotoxicity (ADCC) which is absent in *in vitro* system [19]. Since EGFR plays a significant role in CRC, the ability of its ligand to trigger the downstream signal in KRAS mutant cells was examined. EGF triggered both Akt and ERK phosphorylation in HCT116 cells and induced ERK activation in SW480 cells (Fig. 1B), indicating that KRAS mutation doesn’t fully take over the ligand-mediated ERK activation and also impling the significance of EGFR in KRAS mutant cells. Moreover, pretreatment with HDAC inhibitors, TSA and SAHA, disrupted the EGF-stimulated ERK and Akt phosphorylation in HCT116 cells and ERK phosphorylation in SW480 cells (Fig. 1C). Since HDAC inhibitors blocked both Akt and ERK phosphorylations, the very proximal component of EGF signaling might be targeted by HDACi. Therefore, the expression of EGF receptor was firstly examined. After treatment with TSA, the expression of EGFR was decreased in HCT116, SW480, and HT29 cells. To identify whether this is a common phenomenon, cells originated from different organs were used. After treatment with TSA, the reduced EGFR expression was also seen in human skin (A431) and breast (MDA-MB468) cancer cells (Fig.1D).

**Figure 1:** HDAC inhibitor disrupted the EGF signaling in KRAS mutant colon cancer cells. (A) HCT116, SW480, WiDr and HT29 cells were maintained in DMEM with 1 mg/ml glucose and treated with 0.1, 1, 10 µg/ml cetuximab or 1, 3, 5 µM SAHA the cell survival was measured by MTT assay after 48 hours treatment (B) HCT116 and SW480 cells were serum-starved for 24 hours and then stimulated with 1 µM EGF for, 1, 5, 15, 30 and 60 minutes. (C) HCT116 and SW480 cells were pre-incubated with 0.5, 1 µM TSA or 5 µM SAHA for 24 hours and then stimulated with EGF for 5 minutes. (D) HCT116, SW480, A431 and MDA-MB468 cells were treated with 1 µM TSA for 24 or 36 hours Whole cell lysate was prepared and subjected to western blot analysis with antibodies specific for phospho-Akt, phosphor-ERK, Akt and Erk.

### HDAC inhibitors reduce the expression of SGLT1 and decrease the intracellular glucose

In addition to EGF signaling, EGFR has been reported to be involved in the glucose transport by associating and stabilizing the active glucose transporter, SGLT1 [13], [20]. Since the expression of EGFR was reduced by HDACi in CRC cells, the levels of SGLT1 expression and intracellular glucose in response to HDACi were also examined. As expected, TSA reduced the SGLT1 expression (Fig.2A) and the intracellular glucose concentration (Fig. 2B). Glucose replenishment retained the intracellular glucose (Fig. 2C) and rescued cells from the TSA-induced cell death (Fig. 2D). These data suggested that the loss of EGFR and its partner, SGLT1, might be involved in the cytotoxic effect of HDAC inhibitors.

**Figure 2:** HDAC inhibitor reduced the expression of SGLT1 and decreased glucose uptake. (A) HCT116 cells were treated with 1 µM TSA for 24, 36 or 48 hours. Whole cell lysate were prepared and subjected to western blot analysis with antibodies specific for SGLT1, EGFR and Actin. (B) Cells were cultured in DMEM with 1 mg/ml and treated with 1 µM TSA for 24 hours. The glucose content was measured as described in material and method (Triplicate samples were used in each group. The asterisk indicates a significant difference with p<0.05. Error bars indicate mean ± SE.) (C) Cells were cultured in DMEM with 1 mg/ml or 4.5 mg/ml glucose and treated with 1, 3 or 5 µM TSA for 24 hours. The glucose content was measured. (D) Cells were cultured in DMEM with 1 mg/ml glucose and treated with 1 or 3 µM TSA. After 24 or 48 hours of treatment, the glucose was adjusted to 4.5 mg/ml. The cell survival was measured by MTT assay after 72 hours treatment with TSA. Results were expressed as mean ± SE of three independent experiments performed in triplicate.

### Loss of EGFR is implicated in HDAC inhibitor-mediated cytotoxicity

HDAC inhibitors are shown to exert antitumor activity by arresting the cell cycle and triggering apoptosis [15]. Consistently, SAHA increased sub-G1 population from 7.72% to 17.23% and G2/M population from 16.6% to 24.4% (Fig.3A). To elucidate the role of EGFR in the antitumor activity of HDACi, cells were transfected with myc-EGFR and then treated with SAHA for 24 hrs. Overexpression of myc-tagged EGFR decreased the sub-G1 population and G2/M population (Fig.3A). SAHA-induced p21 expression was also attenuated by the ectopic expression of EGFR (Fig.3B). These data indicated that SAHA-reduced EGFR expression contributed to the SAHA-induced apoptosis and cell cycle arrest.

**Figure 3:** Loss of EGFR contributed to HDAC inhibitor-mediated antitumor effects. (A) HCT116 cells were transfected with Myc-EGFR as well as its vector control and transfected cells were treated with 5 µM SAHA for 24 hours. Cells were fixed by 70% ethanol and stained with propidium iodide, and fraction of cell cycle was analyzed by flow cytometer. (B) HCT116 cells were transfected with Myc-EGFR as well as its vector control and the transfected cells were treated with 5 µM SAHA for 24 hours. Whole cell lysate were prepared and subjected to western blot using Ab specific for EGFR, Myc, p21 and tubulin.

### HDACs are implicated in the transcription of EGFR

Since the amount of EGFR protein is reduced after treatment with HDACi, the EGFR gene transcription was examined. The mRNA level of EGFR was decreased dramatically after treatment with TSA and SAHA (Fig.4A), suggesting HDACi transcriptionally downregulate EGFR expression. This effect was further confirmed by EGFR reporter assays. Our result showed that TSA and SAHA significantly decreased the EGFR promoter activity (Fig.4B upper panel). It has been reported that HDACi decreased the EGFR mRNA stability in ER-negative human breast cancer cells [21]. Therefore, the stability of EGFR mRNA was examined. The *de novo* transcription was stopped by actinomycin D and the EGFR mRNA was measured by real-time PCR. The slope of EGFR mRNA degradation didn’t show a significant difference between basal and TSA treatment (Fig. 4B lower panel), suggesting that HDACi didn’t affect the degradation of EGFR mRNA in colorectal cancer cells. To further elucidate the involvement of HDACs in the transcription of EGFR, myc-tagged HDAC1, HDAC2 or HDAC3 was ectopically expressed in HCT116 cells, and EGFR mRNA was measured by RT-PCR. An increase of EGFR mRNA was found in all these HDAC-expressing cells (Fig. 4C upper panel). Conversely, knockdown of HDAC1, HDAC2 or HDAC3 by shRNA reduced the expression of EGFR protein (Fig.4C lower panel). These data indicated that class I HDACs are crucial for EGFR expression. The positive correlation between EGFR and HDAC3 expression was also observed in fourteen pairs of human colon tumor and adjacent normal tissues (Fig. 4D).

**Figure 4:** HDAC is involved in the regulation of EGFR transcription. (A) HCT116 cells were treated with 1 µM TSA or 5 µM SAHA for 1 and 8 hours. Total RNA (2 µg) was used for RT-PCR and Real-time PCR as described. (B, upper panel) Cells were treated with 1 µM TSA or 5 µM SAHA for 6 hour, then transfected with EGFR-Luc. Luciferase activities were measured as described under “Material and Method”. (B, lower panel) Cells were treated with 1 µM TSA for 4 h before RNA synthesis was stopped by actinomycin D (5 µg/ml) for 0, 2, 4 or 6 h. RNA was prepared at indicated time points following the addition of actinomycin D and levels of EGFR mRNA were measured by real-time PCR. (C, upper panel) Cells were transiently transfected with Myc-tagged HDAC1, 2 or 3, respectively and total RNA (2 µg) was used for RT-PCR to detect the EGFR mRNA level. (C, lower panel) Cells were transfected with shLuc, shHDAC1, shHDAC2 or shHDAC3 by lentivirus as described under “Material and Method”. Cell lysates were harvested on day 5 after transfection and then subjected to western blot analysis with antibodies specific for EGFR, HDAC1, HDAC2 and HDAC3. (D) Lysates of paired human normal and malignant colon tissues were subjected to western blotting using anti-EGFR, anti-HDAC3 and anti-Actin antibodies. The correlation between EGFR and HDAC3 expression levels was evaluated by correlation coefficients.

### SP1 is essential for EGFR transcription and HDAC inhibitor disturbs the binding of SP1 to EGFR promoter

There are several SP1 binding sites on the EGFR promoters and our previous studies showed that HDACi affects the binding of SP1 to ADAMTS1or p21 promoters [22], [23]. Therefore, SP1 may participate in the HDACs-mediated EGFR expression. Indeed, inhibition of SP1 by mithramycin A (MTM) and siRNA significantly decreased the EGFR expression (Fig.5A). Furthermore, MTM drastically reduced the EGFR promoter activity (Fig.5B), indicating the critical role of SP1 in EGFR gene transcription. The binding of SP1 to the EGFR promoter is further examined by chromatin immunoprecipitation (ChIP). Five primer pairs (A, B, C, D and E) were designed to evenly cover the regions (−1,200 to +1,000 bps) around transcription start site (Fig.6A). Our data showed that the binding of SP1 to regions C and D was significantly decreased after treatment with SAHA (Fig.6B). Furthermore, the acetylation of Histone H3 and H4 on EGFR promoter was largely reduced, especially in the regions nearby transcription start site (Fig.6B). The status of histone methylation such as H3K4Me2, H3K9Me3 and H3K27Me3 was also examined. SAHA didn’t change the residence of these methylation markers on EGFR promoter despite of enriched H3K4Me2 was found (Fig.6B and data not shown). Since the acetylation of histone H3 and H4 dropped dramatically after HDAC inhibition, the occupancy of histone acetyltransferase (HAT) or HDAC on EGFR promoter was examined. Our result showed that the recruitment of CBP to region D was significantly decreased by SAHA (Fig.6B). Interestingly, the binding of HDAC3 to the region D was attenuated, too (Fig.6B). These data showed the dissociation of SP1, CBP and HDAC3 from EGFR promoter at the same time (Fig.7), implying that these proteins may influence each other and affect their binding to the EGFR promoter.

**Figure 5:** SP1 is essential for the EGFR transcription. (A) Cells were treated with 1 µM Mithramycin A (MTM) for 18 or 36 hours, then the total cell lysate were prepared. Cells were transfected with 0, 400 or 800 pmole SP1 siRNA, then the total cell lysates were prepared and subjected to western blot analysis with antibodies specific for EGFR and SP1. (B) Cells were transfected with EGFR-Luc and then treated with 0.1, 1 or 5 µM Mithramycin A (MTM) for 16 hours. Luciferase activities were measured as described under “Material and Method”. The results were normalized to the Renilla luciferase activity and expressed as the mean ± SE. For three independent experiments performed in triplicate.

**Figure 6:** The epigenetic alteration on EGFR promoter. (A) Illustration of the EGFR promoter and the ChIP primer. (B) Cells were treated with SAHA for 8 hours, then fixed, sonicated and subjected to Chromatin Immunoprecipitation using Ab specific against SP1 and acetylated histone H3. Histone H4 acetylation H3K4 dimethylation, CBP and HDAC3 on EGFR promoter was measured by ChIP assays as described under “Material and Method”.

**Figure 7:** Schematic diagram of EGFR promoter in the basal state or treatement with HDACi. In the basal state, HDAC3, CBP and SP1 were both recruited to the promoter region and responsible for the transcription of EGFR (A). While treated with HDACi, the complex of HDAC3, CBP and SP1 were disrupted and dispersed from EGFR promoter, leading to the inactivation of EGFR transcription (B).

## Discussion

EGFR and HDAC have been reported to be overexpressed in colorectal and various cancers [1], [15]. However, their relationship is not well-characterized. In this study, we showed that HDAC inhibitors (HDACi) were able to disrupt the EGF-signaling in colon cancer cells. EGFR expression in these cells as well as other origins such as epidermoid (A431) and breast (MDA-MB468) was decreased by HDACi, suggesting the potential of HDACi to treat EGFR overexpressing cancers. HDACi also reduced the expression of an active glucose transporter, SGLT1, and thereby suppressed the glucose uptake of colon cancer cells. More in-depth, we showed that SAHA induced the dissociation of SP1/CBP/HDAC3 from the regions around EGFR transcription start site where the histones became hypoacetylated. Our data indicated that the HDAC inhibitors could serve as a single agent to block EGFR and HDAC, two critical factors in CRC cells, and may provide a more effective therapy for a broader range of indication.

Most solid tumors reside in a hypoxic environment and prefer the anaerobic glycolysis rather than aerobic glycolysis, converting glucose to lactate and produce fewer ATP with less oxygen consumption. Therefore, the glucose uptake is frequently enhanced in tumors by overexpression of glucose transporters, such as GLUT1 and SGLT1 [24]. Unlike GLUT1 that transports glucose passively, SGLT1 uses the electro-chemical sodium gradient to transport glucose against the internal concentration gradient. SGLT1 is expressed in human colon cancers, pancreatic cancer, lung cancer and neoplastic lesions of head and neck [25]–[29]. It is found to be stabilized by EGFR, and knockdown of EGFR decreases the SGLT1 expression and glucose uptake [13]. Our data also showed that HDACi-mediated loss of EGFR, and the concurrent reduction of SGLT1 expression and glucose uptake would eliminate the overall pro-survival functions of EGFR.

Several studies show the inhibitory effect of HDACi on EGFR expression in human cancers. For example, FK-228, a depsipeptide HDAC inhibitor, is reported to decrease the expression of EGFR in lung cancer cells [30]. SAHA decreases the levels of EGFR in ER-negative breast cancer cells via mRNA destabilzaiton [21]. More recently, inhibition of HDAC6 is found to enhance the endocytosis of EGFR through increasing tubulin acetylation [31], [32]. In this study, we demonstrated that both EGFR mRNA and its promoter activity were inhibited by HDAC inhibitors in colon cancer cells, indicating that the *de novo* synthesis of EGFR was transcriptionally inhibited. EGFR promoter is characterized with GC-rich, and TATA-less, and harbors multiple specificity protein 1 (Sp1) binding sites [33]. In addition to SP1, several transcription factors, such as AP-1, p53 and c-Jun, also participate in the EGFR transcription [34]. SP1 has been reported to regulate the basal EGFR promoter activity [35]. We showed that inhibition or knockdown of SP1 could decrease the promoter activity and protein expression of EGFR, emphasizing its crucial role in EGFR expression.

SP1 has been reported to be regulated by several post-translational modifications, including phosphorylation, acetylation, ubiquitination and sumoylation [36]. It is acetylated by p300 and deacetylated by HDAC [37]. Although acetylated SP1 could increase the transcription of GC-box-dependent genes [37], accumulating data also show that acetylation of SP1 decrease the its transcriptional activity. For example, SP1 acetylation by HDACi reduces its ability to regulate 12(s)-lipooxygenase (12S-LOX) expression. Ectopic expression of SP1 mutant, which cannot be acetylated at lysine 703, increases 12S-LOX transcription, and deacetylation of SP1 is also required for the transcription of COX-2 [38], [39]. Our previous studies show that HDACi affects the binding of SP1 to ADAMTS1 promoter and the association of SP1 and CBP on p21 promoter [22], [23]. SP1 on EGFR promoter might be affected by HDACi as well. Indeed, SP1 was dissociated from EGFR promoter after treatment with HDACi, implying that acetylation may decrease the binding of SP1 to the EGFR promoter. Surprisingly, the histones on EGFR promoter became hypoacetylated. This could be explained by the concurrent dissociation of CBP, the histone acetyltransferase (HAT).

HDACi is reported to induce G2/M growth arrest as well as G0/G1 arrest in colorectal cancer cells, and the HDACi-mediated growth arrest consistently involves p21 induction [40]–[43]. In HCT116 cells, p21 is induced and the cell cycle is arrested in G2/M phase by silencing class I HDACs, especially HDAC3 [17]. Consistently, we found that SAHA induced p21 and G2/M arrest and re-expression of EGFR could alleviate these events. HDAC3 has been reported to be maximally expressed in the proliferative compartment in mouse colon. Knockdown of HDAC3 induced a greater magnitude of G2/M and S phase arrest than that of HDAC1/2, suggesting that HDAC3 is more significant than HDAC1/2 in colon cell proliferation [17]. HDAC3 is a component of the NCoR-SMRT co-repressor complex, which is distinct from repressor complexes containing HDAC1 and HDAC2 (Sin3A and NuRD) [44], indicating the specific roles of HDAC isoform in gene repressing. In contrast, knockdown of HDAC1, 2 or 3 decreased the EGFR expression in varying degree, indicating that they share functional redundancy on promoting EGFR transcription. Ectopic express HDAC3 induced a greater magnitude of EGFR mRNA and a positive correlation between EGFR and HDAC3 expression in colon cancer patients. Therefore, HDAC3 may be most essential in EGFR transcription.

Association of HDACs with gene promoters are traditionally considered to repress transcription and HDAC is thought to reactivate the silenced genes [45]. However, HDACi is also reported to decrease the expression of thymidylate synthase, vascular endothelial growth factor (VEGF), basic fibroblast growth factor (bFGF) and endothelial nitric oxide synthase (eNOS) [46]–[48]. It is suggested that gene transcription primed by H3K4 methylation requires the dynamic cycle of histone acetylation and deacetylation by transient HAT/HDAC binding [49]. In this study, we found that EGFR promoter was enriched with H3K4 di-methylation, suggesting that EGFR gene transcription may be primed by H3K4 methylation. HDAC3 and CBP were both associated with EGFR promoter and concurrently dissociated after treatment with HDACi, implying that dynamic HAT/HDAC binding is occurred. Since CBP and HDAC3 are unable to directly bind gene promoter, SP1 may serve as a bridge between CBP/HDAC3 and EGFR promoter (Fig. 6A). HDACi may induce SP1 acetylation and leads to its dissociation from EGFR promoter, which disrupts the dynamic binding of HDAC3 and CBP (Fig. 6B). Taken together, our results showed that the SP1, HDAC3 and CBP were all dissociated from EGFR promoter after SAHA treatment, suggesting their functional relevance on EGFR transcription.

It has been reported that HDAC inhibitors synergize with 5-FU *in vitro* and *in vivo* to treat colon cancer through downregulation of thymidylate synthase, the 5-FU target enzyme [46]. Combination of 5-FU with SAHA has recently entered phase I/II trial to treat CRC [18], [50]. Inhibition of MAPK and Akt signaling by AEE788, a multiple receptor tyrosine kinases inhibitor, synergistically potentiates HDAC-induced apoptosis in a broad spectrum of cancer cell lines [51]. Recently, a new compound, CUDC-101, which inhibit the activity of both EGFR and HDAC, is demonstrated to have powerful anticancer activity [52]. These reports strengthen the rationale of concurrent inhibition of EGFR and HDAC in cancer therapy. In this study, we showed that HDAC inhibitor alone is able to block EGFR transcription as well as HDAC, and may provide a hint for superior strategy of colorectal cancer therapy.
